# Remote Ultrasound Scan Procedures with Medical Robots: Towards New Perspectives between Medicine and Engineering

**DOI:** 10.1155/2022/1072642

**Published:** 2022-02-11

**Authors:** Maide Bucolo, Gea Bucolo, Arturo Buscarino, Agata Fiumara, Luigi Fortuna, Salvina Gagliano

**Affiliations:** ^1^Dipartimento di Ingegneria Elettrica Elettronica e Informatica, University of Catania, Italy; ^2^IASI, Consiglio Nazionale Delle Ricerche (CNR), Roma, Italy; ^3^Azienda Ospedaliera per l'Emergenza Cannizzaro, Catania, Italy; ^4^Regional Referral Centre for Inborn Errors Metabolism, Pediatric Clinic, Department of Clinical and Experimental Medicine, University of Catania, Italy

## Abstract

**Background:**

This review explores state-of-the-art teleoperated robots for medical ultrasound scan procedures, providing a comprehensive look including the recent trends arising from the COVID-19 pandemic.

**Methods:**

Physicians' experience is included to indicate the importance of their role in the design of improved medical robots. From this perspective, novel classes of equipment for remote diagnostics based on medical robotics are discussed in terms of innovative engineering technologies.

**Results:**

Relevant literature is reviewed under the system engineering point of view, organizing the discussion on the basis of the main technological focus of each contribution.

**Conclusions:**

This contribution is aimed at stimulating new research to obtain faster results on teleoperated robotics for ultrasound diagnostics in response to the high demand raised by the ongoing pandemic.

## 1. Introduction

Advanced robotics play a fundamental role in performing complex and sensitive tasks related to teleoperated medical procedures. To ensure safe and reliable operations under both the remote guidance of a physician performing the medical procedure and a completely automated procedure, a suitable level of performance regarding the precision of the robotic system must be reached, and precision is affected by communication delays, sensor capabilities, and user interfaces. These characteristics make the design of such systems a multidisciplinary and emerging topic that encompasses instrumentation, measurement, telecommunication, and robotics engineering, all of which are necessary to provide innovative engineering solutions.

In this paper, we aim to review the recent literature on the design of advanced equipment for teleoperated medical ultrasound scan procedures, a simple but effective medical procedure that may save lives in difficult environments and remote areas if promptly performed by an expert, who is likely located far from the patient. Unlike other reviews in the literature [1] that are oriented toward specific medical applications, this contribution provides a comparative collection of the technological results presented in an organized manner in order to provide a complete overview of existing equipment, focusing on the main topics and solutions and highlighting current limitations.

The design of remotely operated medical devices must occur within a wider framework of emergent technologies. In fact, such topic requires a comprehensive global perspective, covering various multidisciplinary areas and their relevant advanced topics. Therefore, this review is aimed at establishing a wider view regarding advanced projects and current research.

First, a macroscale analysis of the complex engineering aspects and concepts involved is performed. From a more general perspective, we obtain a precise collocation of the particular problems to be solved. Furthermore, a clustered review of state-of-the-art teleoperated ultrasound scan techniques is proposed. Finally, we discuss various innovative aspects currently under evaluation, paving the way for future research aimed at improving the efficiency of current solutions bearing in mind physician experience.

The scientific contributions reviewed in this manuscript present solutions that range from preliminary simulations and prototypes to medical solutions already available to physicians. Therefore, patient management differs depending on the solution. In particular, we highlight cases in which the presence of technical or sanitary staff is needed at the patient location, with some cases in which the staff must be fully trained and other systems that do not require special skills to position the medical robot. When appropriate, we specify the patient management conditions in the discussion regarding each solution.

It is worth noting that the year 2020, with the outbreak of a massive pandemic, highlighted the importance of designing low-cost telemedicine solutions and the need for advanced teleoperated equipment. Efforts should be dedicated every day to new research that provides the highest benefits to patients by improving the quality of physicians' experience using remote techniques when they are prevented from being in direct contact with a patient. Therefore, this contribution aims to stimulate new research to obtain further results in the use of teleoperated robotics for ultrasound diagnostics.

## 2. System Engineering Point of View

A constructive approach to modeling has led the development of human studies toward a universe consisting of algorithms and technologies over the past century, thus conceiving and developing systems that reach beyond a single purpose. The theory of complexity provides an approach for researchers from different disciplines to share knowledge to conceive solutions to large-scale problems beyond the reductionist approach. Biomedicine and biomedical engineering are emerging examples of this approach. Engineering, physics, and medicine have been connected in an organized and standardized way to develop complex engineering design procedures applied to medicine [2].

The interplay between medicine and technology can be discussed from a wide range of viewpoints and applications, as it falls within the wider framework containing topics such as human-machine interaction. In this review, we provide a system engineering point of view on a specific branch of biomedical robotics—teleoperated medical robots for ultrasound scan procedures—as this branch represents the basis of new paradigms for modern medicine diagnostics.

Such a topic involves the interaction between the robot and the physician, especially when a physician is at a different location with respect to the patient. In these cases, the physician should be able to experience the same physical perception as if directly in contact with the patient. To this end, particular equipment must be available to guarantee a high degree of accuracy, a high level of safety, and a fast diagnosis [3, 4].

To demonstrate the importance of this topic, consider a naive Google search, as summarized in Figure 1(a). Searching for *human-machine interaction*, Google produces 269,000,000 items in 0.57 seconds, *remote robotics* appears 92,600,000 times, *new medical technological paradigms* 104,000,000 times, and *telemedicine* or *telehealth* 19,200,000 times.

Including *remote ultrasound medicine*, we obtain 45,200 results. In Figure 1(b), the importance of this latter topic is emphasized by comparing it to the other topics at the border between robotics and medicine. The figure shows that ultrasound scan procedures performed by teleoperated medical robots cover an important slice in the cluster containing meta-technological areas of advanced complex systems.

Even before the outbreak of the COVID-19 pandemic, the request for medical remote operations has been increasing every year, the obvious advantage being that the operator can provide life-saving procedures in remote areas without being physically present. The effect is that the literature on teleoperated robotics for ultrasound scan procedures involves different topics and technological solutions.

Performing a search over SCOPUS for scientific contributions on the topic of remote ultrasound, approximately 2,191 items were retrieved. These contributions can be classified according to a system engineering perspective based on the following items:

- Systems: contributions related to the design of comprehensive, often commercial, apparatuses
- Control: papers including control solutions to improve precision of the robot and to increase safety of operations
- Mechanical characterization of tissues: contributions related to the modeling and characterization of human tissues properties to improve robot control
- Human-robot interface and sensors: papers aimed at proposing solutions to improve the experience of the physician in performing the remote operations, including sensing capabilities
- Vision and image processing: algorithms to improve the visual perception of the remotely operating located physicians
- Training and current trends: description of educational campaigns to improve the usability and effectiveness of remotely operated ultrasound scan procedures

These items represent the more intriguing technical aspects related to novel robotic systems for medical procedures in general, but for remote ultrasound scan procedures in particular, as they cover all the technological problems related to this type of procedure. In addition to considering complete systems designed for this purpose, it is interesting to analyze the different solutions related to the specific problems involving modeling and characterization of tissues, sensor capabilities, and image processing techniques needed to improve the safety, reliability, and performance of fully autonomous systems. Finally, training is fundamental in preparing forthcoming generations of physicians for an occupation in which the presence of robotic systems will considerably increase over the next few years.

The bar plot in Figure 2 shows the fraction of the 2,191 Scopus results in which each item is addressed. It is evident that the control problem is the most challenging topic, followed by the mechanical characterization of tissues, and finally, sensing devices. The trend for each item can be obtained from Figure 3, where the number of publications per year related to each topic is reported. Besides being the most considered topic, control continues to grow, while the trend involving scientific papers related to tissue properties has reached a steady value. In particular, the trends related to vision systems have increased over the past two years with respect to training and education. This latter topic is fundamental, as it is arguably directly linked with the outbreak of the COVID-19 pandemic.

## 3. Robotics for Remote Ultrasound Scan Procedures

In this section, we review the fundamental literature involving teleoperated ultrasound scan procedures. The contributions will be reported according to the classification presented above.

### 3.1. Systems

Consider the topic of teleoperated systems beginning with commercial and comprehensive solutions currently available, as discussed in the literature.

Developing novel setups that can address the problem of teleoperated ultrasound scan procedures involves many engineering and physics problems [5]. One of the primary issues in remote medicine and robotics for remote ultrasound scan procedures is the communication between the robot and the physician. In fact, to date, there are no standard protocols that guarantee secure connections explicitly for medical purposes. The lack of standard protocols makes it difficult to directly compare the different approaches. In the following section, we highlight the weaknesses and strengths of each solution.

One common problem in systems for teleoperated medical procedures is the delay that occurs during the transmission of control signals. The use of the Internet to share information between a remote (where the patient and the robot are located) and a local (where the physician operates) station does not guarantee stable latency. The control of robotic arms is often performed through user-defined software packages. In some cases [6], synchronization between the reference signal and the output of the system is not ensured because unavoidable delays are not integrated in the control design. In contrast, other applications, specifically designed for surgery [7] and patient rehabilitation [8], are able to provide higher accuracy and reliability despite communication delays. In [7], a 10 Mbps bandwidth was adopted (6 Mbps was actually sufficient) to ensure the capability to perform an action with a maximum delay of 1 s. It should be mentioned that this setup relies on a dated infrastructure, and current technologies may improve system performance. Regarding wireless operations, in [9], a solution based on 4G was described, leading to a video delay on the order of 100 ms.

Another problem is the operator physical experience. Systems designed specifically to improve the experience of physicians have been proposed [10]. They focus on reducing or preventing musculoskeletal disorders for physicians, which are related to the operation of the virtual ultrasound probe, such as holding transducers in awkward positions for long time intervals [11, 12]. In [13], an ultrasound robotic system based on the commercial robot UR5 was introduced with the aim of reducing the strain on radiologists shoulders. From a different perspective, the experience of the operator can be improved in terms of the sensory feedback perceived during operations. A system specifically intended for tele-echography, named TER [9], includes different sensors [14], such as force sensors, to provide force feedback during the control action to improve the probe degree of freedom, allowing the physician to provide different pressures on the remote patient body.

The solution reported in [13] exploits a master-slave configuration, including a strict safety protocol acting over three distinct layers, i.e., hardware, software, and user interface. The application is designed to be operated either locally or remotely, thus introducing higher reusability and configurability. Data transmitted from the slave to the master station include forces, torques, and velocity; thus, haptic control can be implemented at the master station. This solution has become a standard for teleoperated ultrasound scan procedures in recent years.

The system presented in [15] was conceived to provide high-quality image feedback to the remote operator, providing a high success rate in a clinical study. In particular, focus was on correct and timely diagnosis involving obese patients. Faults in the proposed system were linked to poor echogenicity of the pancreas and gallbladder, and to the presence of edema, preventing proper imaging of the deep veins in the leg.

The MELODY system [16] is a commercial robotized ultrasound diagnostic product. Using this system, the expert can manipulate a *dummy probe*, similar to the real probe, allowing rapid control of the robotic arm from a remote location. The main advantage of this technology with respect to the other discussed solutions is that its functionality is guaranteed even with a limited Internet bandwidth (2 Mbit/s), allowing it to be fully operational in rural areas. Moreover, on the patient side, a healthcare professional with no ultrasound skills can assist the imaging expert by positioning the robotic arm over the patient.

In the system proposed in [17], a tele-robotic arm was also used to perform renal biopsies using ultrasound. The procedure is performed under guidance from a radiologist remotely controlling the robotic arm. In 1999, the Hippocrates project [18] led to a robot-assisted ultrasound diagnostic system created to prevent cardiovascular diseases.

The systems discussed in this section have the common characteristic of providing comprehensive solutions for high-quality teleoperated ultrasound scan procedures. Some are designed for specific tasks and therefore require the involvement of specialists and skilled technical staff. Other commercial solutions, such as TER, UR5, and MELODY, provide complete solutions that can be used with minimal training. Readers can refer to [19] for a complete review of minimally invasive robotics solutions.

The main features and limitations of the reviewed approaches are summarized in Table 1.

### 3.2. Control

The specificity of the control problem in teleoperated medical procedures requires the design of innovative solutions and approaches. Because of the time delays introduced by the communication network between local and remote stations and the uncertainty of the patient body model, a robust adaptive control scheme with predictive action must be implemented [21, 22]. Hence, the robustness of the control scheme must be evaluated accurately.

Force and position control systems must be designed according to strict and critical conditions typical of medical procedures. In this regard, the approach proposed in [23] is notable, where a control framework based on the construction of a confidence map is intended to optimize ultrasound image quality. A different approach based on a direct real-time measurement of the pressure using a strain sensor and probe combination is discussed in [24]. The application of genetic algorithms for the determination of the gains associated with a control action has been discussed in [25], leading to an improvement in positioning precision and a decrease in the induced pressure.

The interplay between control strategies and tissue response is, therefore, a critical item in the design of medical robots. Beyond the ultrasound scan, this aspect has been explicitly considered in [26, 27], where a control action based on accurate tissue modeling allows for teleoperated needle insertion.

Recently, a software framework to simulate the positioning of a teleoperated medical robot was proposed [28]. This framework proved to be useful in testing innovative control actions and in training physicians in the use of advanced teleoperated robotic systems.

Particular focus is being applied to the problem of force-feedback control, that is, the possibility of providing remote tactile information regarding the mechanical interaction between the teleoperated probe and patient tissues.

The study presented in [29] is notable, where the analysis of the relationship between physicians and user interfaces involving ultrasonography devices was carried out, concluding that virtual reality alone is not sufficient to reproduce the effectiveness of a locally performed scan. In ultrasound scan procedures, not only the image provides information but also the direct tactile information process. Therefore, the importance of force feedback is not only limited to assisting the control action of the robotic arm but also allows the physician to feel a physical response from the probe. Such feedback will provide a fundamental insight that is still missing in all the robotics solutions discussed previously.

According to this idea, the physician should use an artificial body [30] with a probe emulating the use of the sonograph on the real patient's body. The ideal condition would be the use of an artificial body that, by means of distributed actuators, creates feedback that the operator can feel as a tactile force [31]. The main issue is that there is currently no artificial body on the market that meets these requirements. A possible solution is the use of a more readily available product, already used in the medical field, such as a desktop haptic interface that allows the operator to receive force feedback from the patient and provides a simple interface.

The inclusion of force-feedback control represents a significant improvement in this type of medical practice, although specific control problems arise.

In [11], a pioneer study on the advantages of adopting control actions based on force feedback was shown and described, and the first attempt to implement this type of control was a teleoperated mobile ultrasound scanner for real-time image acquisition and diagnosis based on six degrees of freedom [15]. In this application, a force sensor provides information regarding the contact force between the probe and the patient skin. Moreover, a strategy to stabilize the ultrasonic probe reported in [32] was based on the adoption of force feedback to determine the specific pressure applied to patient tissues. Indeed, tactile sensing technologies emphasize the role of sensing information in biomedicine [33].

A recent study [34] envisaged the realization of a novel force-feedback device based on an artificial body, implemented using electromechanical structures based on viscoelastic materials [35], in which air chambers filled using a controlled air flux were considered. This implementation provided human-like tactile feedback to the physician during the ultrasound scan procedure.

The reviewed results are schematized in Table 2 highlighting the control features and their limitations.

### 3.3. Mechanical Characterization of Tissues and Calibration

Research on innovative solutions must also rely on the capability to model human tissues and their mechanical characteristics. With regard to the modeling of body-like structures, the use of specific materials is fundamental. From the point of view of artificial bodies, a model using a polyvinyl chloride (PVC) phantom, specifically oriented to robotics and robot interaction, is fully described in [36], whereas an interesting study on biomechanical models of myocardium [37] provides insights into the possibility of realizing active artificial bodies for advanced remote medical diagnostics.

In addition, in the context of artificial bodies, extensive use of tissue-mimicking materials for training physicians and ultrasound scan operators is discussed in [38]. A similar approach was proposed for the real-time calibration of ultrasound probes in [39], where a phantom based on piezoelectric material with multiple active points is introduced to improve the accuracy and precision of the probe. A phantom to obtain spatial calibration of a remotely operated ultrasound probe is discussed in [40], where a spatial reconstruction of the probe position is performed by applying a Gaussian mixture model approach that provides higher accuracy, although it increases the mathematical complexity of the calibration procedure.

The models discussed in this subsection have the common characteristic of being tailored to the specific tissue they mimic. Their capability to reproduce the actual mechanical response of a given human tissue is evident, but the lack of a general framework to realize physical devices mimicking different parts of the human body currently prevents their broader diffusion. The possibility of considering viscoelastic programmable devices, such as those envisaged in [34], or with internal artificial vessels based on microfluidic networks [41], is worth investigating in detail to overcome the limitations of current approaches.

A comparison on the main features and limitation of the reviewed contributions is reported in Table 3.

### 3.4. Human-Robot Interface and Sensors

The problem regarding the human-robot interface deserves deeper investigation, as it represents a crucial step toward improving both research and operation of medical robots in general, and has particular relevance for teleoperated ultrasound scan devices. The fact that the physicians are distant from the patients implies that they are not able to directly *feel* the body reaction, something that is required even for highly skilled medical personnel. To improve the capability to compensate for the separation between the operator and the patient, the interface with the medical robot must be enhanced.

The use of a haptic device to control the robot through an intelligent probe scaling the forces to allow a more ergonomic holding position was evaluated in [11]. An interesting point made in this study is that the system is realized using low-cost components, and its interface is compatible with commercial robots.

The system in [11] has several modes of operation: *operator control*, where the system operates in the master-slave mode and the information from the probe can be displayed directly with respect to the operator hand; *shared control*, where the operator controls the motion of the ultrasound probe along some degrees of freedom, while the computer controls the motion along other degrees of freedom; *taught control*, where the computer can remember trajectories, thus allowing effortless repeated scans in the same mode. In the master site, the physician can use a manual controller, for example, a joystick that can provide strength feedback to the robot.

In some patients [12, 42, 43], the ultrasound probe used for diagnosis is adapted to perform interventions, for example, to guide needles or other instruments to introduce anesthetics and to perform surgery. The system consists of a master hand controller, a slave manipulator carrying the ultrasound probe, and an associated computer system that allows the operator to remotely position the ultrasound transducer. One of the problems considered was artery examination, which was performed to detect occlusive disease in the left and right common carotid arteries, a major cause of stroke.

A specific and comprehensive review of solutions related to human-robot interfaces in upper limb prosthetics can be found in [44], in which the communication between physician and patient through a video link is fundamental.

Because the technological aspects related to the interactions among physician, patient, and robot are fundamental, both the problem of standardizing engineering solutions [45] and using advanced computer-assisted design technology combined with improved ultrasonic sensors [46] are aspects that must be considered during the design procedure.

A comprehensive review of haptic interfaces for teleoperated medical interventions can be found in [47].

Current efforts lean toward enhancing the portability of the teleoperated device, such as discussed in [48], where an ultrasound scanner for electromyography was realized by combining the two sensing elements using a common interface. In this context, [49] proposed an improvement using miniaturized sensing arrays based on a synthetic aperture approach, which leads to more accurate sensing without increasing the size of the probe.

### 3.5. Vision and Image Processing

A key aspect of teleoperated ultrasound scanning medical devices is the quality of the video flow and of the imaging system.

A measurement system based on photo sensors was proposed in [50] to avoid excessive stress on the patient due to the applied force. The integration of a new-generation ultrasound probe based on optical fiber sensors with a remote-controlled robotic arm was described in [51], providing a solution capable of performing a scan that returns an ultrasound map of an 80 × 80 mm area.

Recently, with the aim of enhancing the information gained from the visual output of an ultrasonic probe, the possibility of exploiting real-time filtering algorithms has been discussed [52]. A comprehensive vision system intended to assist orthopedic surgery was described in [53]. The system consists of the integration of control and image processing systems that encompass novel reliable algorithms and features. These include real-time measurement from ultrasound images fed back to the positioning system, thus increasing the accuracy and safety of a surgical procedure.

Intelligent algorithms based on neural networks have recently been introduced in the analysis and improvement of ultrasound images [54]. These algorithms can extract features of medical interest for a prompt diagnosis from the raw radiofrequency data captured by the ultrasound probe through the use of deep learning techniques and convolutional neural networks. This latter approach was exploited in [55] to improve ultrasound theranostic systems.

An evaluation of the effects of latency in teleoperated ultrasound scan procedures, with particular reference to issues linked with visualization, was carried out in [56], where a novel real-time solution was proposed to overcome the limitations of standard devices.

Moreover, remote probe positioning affects the clarity of the image, such that calibration of the ultrasonic probe must be performed remotely. In [57], a spatial localizer based on sensing magnetic forces was used to calibrate a three-dimensional (3D) tracking system, whereas [58] introduced a strategy based on gradient descent optimization to calibrate an ultrasound probe.

At the boundary between vision and control, the recent work by [59] is notable, where the optimization of an ultrasound scan robot for fetal imaging is presented. The system is designed to guarantee improved safety performance regarding probe pressure and precision to avoid harming the fetus. The results discussed therein are promising, but the system does not have remote-control capabilities.

The solutions discussed in this subsection are mainly research results that are still not compliant with clinical standards. In particular, these proposed solutions should be correctly interfaced with a reliable storage and communication system within healthcare networks based on standards such as Digital Imaging and Communications in Medicine (DICOM) [60] and Health Level 7 (HL7) [61]. Examples of recent DICOM and/or HL7 compliant solutions can be found in [62–64]. By using a KUKA LBR medical robot [65], the authors of [62] proposed a completely autonomous tracking system to improve the focus of ultrasound scan images, storing the image flows following the DICOM standard. In this case, image flows are needed to determine tracking actions. From a different perspective, a DICOM-compliant system designed to merge transrectal ultrasound scans with magnetic resonance imaging was proposed in [63]. Finally, we mention the preliminary results presented in [64] intended to combine artificial intelligence and vision systems for medical purposes by following the HL7 standard to ensure reliable data transfer and data processing.

The main features and limitations of the discussed results are summarized in Table 4, which allows for a direct comparison of the proposed approaches.

### 3.6. Training and Current Trends

Teleoperated ultrasound scan procedures also play a fundamental role in the education of physicians. The use of advanced medical robots provides education either for biomedical engineering studies or for physicians who must be fully trained in their use. In [66, 67], a large-scale program involving rural Australia addressed physician training. A review of general remote medical education in developing countries can be found in [68]. In general, the use of medical robotics as an essential component in medical education [69] is rapidly being assessed.

## 4. Medical Robots for Ultrasound Scan Procedures in the COVID-19 World

Solutions to perform remote medical procedures have gained unprecedented attention in recent years as a consequence of the COVID-19 pandemic outbreak, and the use of medical robots is becoming a fundamental part of modern courses for physicians. In general, medical robotics is becoming a relevant part of physician skills training. Physicians are often prevented from coming in direct contact with infected patients, and even the simplest life-saving procedures cannot always be performed in a timely manner. During the COVID-19 pandemic, a series of studies have addressed this problem and should be mentioned here as future trends for teleoperated medicine [20, 70], even if some solutions are only at a prototype or feasibility study level.

In [71], a novel setup, named MGIUS-R3, is described. It has been conceived as a tool to assist patients with coronavirus by performing remote real-time cardiopulmonary assessment via ultrasound scans. The system is effective because it uses a dedicated 5G communication protocol to ensure stable latency, which guarantees accurate control of the robotic arm and includes a high-quality imaging system. A similar approach is described in [72], but includes a force control loop to allow for different levels of compression of the patient tissue, thus improving the image clarity. The use of reliable 5G communication protocols appears to be fundamental for the solution envisaged in [73] related to a comprehensive software/hardware framework in which data related to patients are fully integrated with robotic equipment, thus remotely performing complete monitoring of infectious patients, thus reducing the need for direct contact.

Follow-up of long-COVID patients also involves continuous monitoring of lung conditions. In [74], a robotic system to perform remote tele-echography to prevent pneumonia is proposed. The key advances of the system are its light weight and the relative ease of the setup phase.

A more specific survey on recent advanced medical and robotic solutions to face COVID-19 related problems can be found in [75].

## 5. Conclusions

Remote diagnostics is becoming a key element of modern medicine in view of the pandemic waves that characterize current times. In this study, we focused on the literature related to use of ultrasound scan procedures operated remotely, showing that the topic involves many points of view and that the different viewpoints can be classified according to a nonreductionist paradigm based on the theory of complex systems.

We performed a direct comparison of the solutions proposed, envisaged, or implemented in different areas related to this broad topic. Moreover, we focused on the key elements that prevent remote ultrasound scan procedures from being as effective as locally performed procedures. In particular, the lack of low-cost artificial bodies that mimic the tissue characteristics of real parts of the human body [30] and the force-feedback signal, already available for control purposes, are not always used to provide the remote operator with the actual physical reaction of the tissue.

The reader can observe the current main limitations of the state-of-the-art from the tables provided in this study. It is clear from Figure 3 that current research trends toward the improvement of control actions, vision systems, and operator training. Although the latter aspect is directly connected to the ongoing pandemic conditions, the need for improvements in control and vision systems is, in our opinion, a convergent goal. Modern and effective control systems are analyzed in view of fully autonomous diagnostic robots [20], that is, systems conceived to interact autonomously with patients and function in the associated environment. Consequently, improvements to on-board vision systems involve two approaches: first, improving the ultrasound scan image quality over remote connections, which may be slow or unreliable, especially in wartime conditions [76] and in nonurban environments, and second, a fully autonomous robot needs an improved vision system to move in different environments under high safety constraints [71].

Recent trends are essentially oriented toward these aspects. Moreover, the increased need for teleoperated diagnostics, linked with the COVID-19 outbreak, is currently pushing the research that should lead to a rapid improvement of available devices. The pandemic scenario along with the desire for long-distance medical diagnosis is thus driving the increased use of teleoperated devices.

The current studies involving state-of-the-art medical robots for ultrasound scan procedures are focusing on advanced technological solutions based on innovative design, thus providing a starting point for continuously improving various systems that will prove useful to biomedical engineering researchers.

In just one year, the demand for devices and solutions for teleoperated diagnostics has increased remarkably, making the topic particularly urgent. This presents various ethical problems regarding the relationship between patients and robotic equipment [77–79]. For a complete review of legal and ethical issues, we refer readers to the comprehensive review by [80]. In the papers discussed in this review related to effective in vivo use, patients are often accompanied by sanitary staff; therefore, any potential negative feelings by the patient are mitigated by providing a human presence (mimicking the presence of a physician) at the location [81].

Furthermore, it is important to highlight the increasing demand for employment positions related to medical robotics engineering. These considerations are leading new generations of engineers toward strict cooperation with physicians in order to find easier, more reliable, low-cost solutions in the field of medical robots for ultrasound scan procedures, as well as in the emerging perspective of the role played by remote medicine and remote activities in modern and future societies. Finally, low-cost medical robots are essential, as they are fundamental tools needed in depressed areas where teleoperated devices can easily perform simple life-saving procedures.

In summary, this review provides a comprehensive framework of the emerging engineering aspects and research trends (as shown in Figure 3) linked to medical applications and procedures performed by (or with the aid of) robotic equipment. This review, together with the study on advanced bioinspired solutions [82] for medial robots, can assist novel generations of biomedical, electronics, and computer science engineers, and physicians to gain information on current trends and drive future research in this strongly multidisciplinary field.

## Figures and Tables

**Figure 1:** (a) Google results obtained for metatechnological areas. (b) Google results for metatechnological areas related to medicine.

**Figure 2:** Relevance of each item within the total number of Scopus results related to remote ultrasound scan systems.

**Figure 3:** Temporal trends of Scopus results published between 2011 and 2021 using the proposed classification.

**Table 1:** Comparison of different complete systems for tele-operated ultrasound scan procedures.

Reference	Main features	Limitations	Clinical/medical applications
Tang et al. [6]	Coordination of heterogeneous master-slave structure	Delays not included in the control law	General applications
Masuda et al. [7]	Wireless tele-echography	Specialized personnel needed to place the robot	General applications
Krebs et al. [8]	Therapy optimization	Specific rehabilitation task	Stroke rehabilitation
Gourdon et al. [9]	High-precision slave system with pneumatic artificial muscles	Limited speed	General applications
Salcudean et al. [11, 12]	Ergonomic interfaces	Lack of 3D image reconstruction	Carotid artery
Mathiasen et al. [13]	Force, haptic, and position control; high real-time performance	Preliminary user interface	General applications
Vilchis et al. [14]	Light-weight autonomous robot	Lack of force feedback	Abdomen
Fjellin et al. [15]	Haptic feedback	No in vivo testing	General applications
Arbeille et al. [16]	Good real-time performance over slower teleconnections	Longer examination sessions	Fetal analysis
Bruyere et al. [17]	Reliable remote operations	Discomfortable setup for the operator	Renal biopsy
Huang et al. [20]	Imitation learning of clinical procedures	Environment scanning performed off-line	Carotid artery

**Table 2:** Comparison of different control strategies.

Reference	Control features	Limitations	Clinical/medical applications
Chatelain et al. [23]	Confidence-drive position control	Simplified ultrasound propagation model	General applications
Skerl et al. [24]	Pressure control	High weight	Abdomen
Kim et al. [25]	Force feedback	Limited force	Thyroid
Abolhassani et al. [26]	Trajectory planning	Slow velocity	Prostate therapy
Li et al. [27]	Trajectory planning	Lack of in vivo testing	Lumbar puncture
Böttger et al. [28]	Dexterity and kinematics	Simulations only	Microcirculation
Filippeschi et al. [29]	User interface including navigation	Remote conditions simulated only	Abdomen
Sénac et al. [31]	Review of pneumatic actuators control	No in vivo testing	Neonatal procedures
Gilbertson et al. [32]	Force and position control	Soft tissues	Muscular systems
Kaminski et al. [33]	Force feedback	Feasibility study	Thyroid diseases
Bucolo et al. [34]	Force feedback	Prototype only	Abdomen
Hadjikov et al. [35]	Model-based control	Simulations only	Abdominal fascia

**Table 3:** Comparison of mechanical characterization of methods for tissues.

Paper	Main features	Limitations	Clinical/medical applications
Haddadi et al. [36]	Improved tissue characterization robustness	Performance decrease at higher robot speed	Artery calcifications
Avazmohammadi et al. [37]	Complete gallery of heart tissue models	Limited analysis of pathological conditions	Myocardium analysis
Dewi et al. [38]	Comparative analysis of heart tissue models	Limited technological aspects	Heart tissue
Zhang et al. [39]	Phantoms based on innovative materials	Midplane detection needed	Abdomen
Wen et al. [40]	Calibration procedure based on tissue identification	Bad conditioning	General applications
Cairone et al. [41]	Detection of microcirculation anomalies	Abstract modeling	Microcirculation

**Table 4:** Comparison of vision and image processing solutions.

Paper	Main features	Limitations	Clinical/medical applications
Nakadate et al. [50]	Reducing fatigue of sonographers and patients	No user interface; lack of object detection algorithms	Abdomen diseases
Colchester et al. [51]	3D tissue reconstruction	Reduced precision for subsurface structures	Vascular system
Geng et al. [52]	Increase of patient safety	Low real-time performance	General applications
Gonçalves et al. [53]	3D bone reconstruction	Limited accuracy and speed	Orthopaedic surgery
Nair et al. [54]	3D feature extraction from raw data	Tested on simplified phantoms	Cysts detection
Igarashi et al. [55]	Detection and tracking of kidneys	Limited detection performance	Tumor lesions tracking
Al-Badri et al. [56]	Real-time remote visualization	Not tested on medical robots	General applications
Pagoulatos et al. [57]	Enhanced calibration for probe position tracking	Need of tissue characteristics knowledge	General applications
Ackerman et al. [58]	On-line self-adaptive calibration	Single calibration method	General applications
Housden et al. [59]	Improved safety features	Probes motion control based on inverse kinematic only	Fetal imaging
Unger et al. [62]	Standardized anatomical structures reconstruction	Higher performance with slower movements	Fibroids and prostate cancer
Moon et al. [63]	Standardized fusion imaging	Tested on phantoms	Prostate biopsy
Pianykh et al. [64]	Standardized AI algorithm implementations	Review of existing solutions	General applications
